The article "Current aspects of multimodal ultrasound liver diagnostics using contrast-enhanced ultrasonography (CEUS), fat evaluation, fibrosis assessment, and perfusion analysis – An update" was retracted in 2025. Reasons: compromised peer review; concerns about the citations; concerns about a third party's involvement.

# Current aspects of multimodal ultrasound liver diagnostics using contrast-enhanced ultrasonography (CEUS), fat evaluation, fibrosis assessment, and perfusion analysis – An update

**DOI:** 10.3233/CH-239100

**Published:** 2023-02-28

**Authors:** E.M. Jung, Yi Dong, F. Jung

**Affiliations:** a Institute of Diagnostic Radiology, Interdisciplinary Ultrasound Department, University Hospital Regensburg, Regensburg, Germany; b Department of Ultrasound, Xinhua Hospital Affiliated to Shanghai Jiaotong University School of Medicine, Shanghai, China; c Institute of Biotechnology, Brandenburg University of Technology, Senftenberg, Germany

**Keywords:** Contrast enhanced ultrasonography (CEUS), fibrosis, perfusion analysis, liver cancer

## Abstract

Current ultrasound multifrequency probes allow both improved detail resolution and depth of penetration when examining the liver. Also, new developments in vascular diagnostics, elastography with fibrosis assessment, evaluation of possible steatosis, and parametric and time intensity curve (TIC) analysis of dynamic microvascularization of the liver with contrast-enhanced ultrasound sonography (CEUS) complement ultrasound-guided diagnostics. State-of-the-art high-resolution technology includes a high frame rate (HiFR) mode for CEUS, fast shear wave measurements with the sound touch quantify (STQ) mode, artifact-free flow detection using HR flow and glazing flow in combination with a special flow-adapted imaging (Ultra Micro Angiography, UMA) and additionally different assessments of possible fatty liver (UltraSound ATtenuation Imaging Technology, USAT). In 50 cases with focal liver lesions, a multimodal liver diagnosis was performed with a still new high-performance ultrasound system as part of the clarification of questions from the university liver consultation and tumor outpatient clinic.

## 1 Introduction

Ultrasound is the most widely available imaging modality worldwide. At the same time, ultrasound imaging is required to be highly detailed and to be able to detect a multitude of morphological and dynamic organ changes as multimodally as possible with one probe. With respect to modern ultrasound techniques, most developments are occurring for improved liver imaging with ultrasound. These include improved vascular ultrasound techniques, various techniques for ultrasound elastography to noninvasively detect the degree of fibrosis, and contrast-enhanced ultrasonography (CEUS) to further clarify unclear findings in B-mode [1–5]. Furthermore, the extent of fatty liver disease has to be detected non-invasively at an early stage [6–8].

To define measurable values, a multiplicity of technical developments have been successfully implemented in high performance ultrasonic devices in recent times [9–12]. In this way, it appears possible to first create a high-resolution B-mode scan with a multi-frequency probe of 1 to 6 MHz with a high level of detail. Strain elastography or shear wave elastography, now also color-coded strain or 2D shear wave elastography and focused point shear wave elastography in the sound touch quantify (STQ) technique can be used to differentiate the degree of fibrosis to cirrhosis and to monitor in the course of various diseases of the hepato-biliary system [13, 14]. Comprehensive modified ultrasound-based liver fat imaging (UltraSound ATtenuation Imaging Technology, USAT) techniques also allow quantification compared to the kidney (HRI+), locally (USAT), or even weighing against additional inflammation.

The article "Current aspects of multimodal ultrasound liver diagnostics using contrast-enhanced ultrasonography (CEUS), fat evaluation, fibrosis assessment, and perfusion analysis – An update" was retracted in 2025. Reasons: compromised peer review; concerns about the citations; concerns about a third party's involvement.

New vascular ultrasound techniques show a significant reduction in artifacts. And with CEUS, quantification of microvascularization can also be done parametrically or as TI analysis in false colors or as dynamical time intensity curves [15–19].

These comprehensive technical ultrasound capabilities still need to be clinically applied and further developed and evaluated in terms of diagnostic capabilities [7, 20]. For example, a new high-end ultrasound system should be used to test assess the extent of steatosis (USAT), vascular tools (Ultra Micro Angiography, UMA) and CEUS perfusion can open up new possibilities on the basis of different cases from the university outpatient liver clinic.

## 2 Material and methods

All examinations were performed by an experienced examiner (>3000 examinations/year, >20 years) using a high-end ultrasound machine (Mindray/Resona R9) with a convex probe from 6 to 1 MHz. Requests for ultrasound examinations were made by the liver outpatient clinic of the university or based on tumor board decisions. Written informed consent was available for CEUS examinations in all cases. CEUS liver diagnostics comply with the EFSUM Guidelines as on-label use [10, 21]. There is also an ethics vote of the local ethics committee (as parts of the DEGUM IV study) [22].

Possible liver lesions were measured in B-mode and macrovascularization was documented with color-coded Doppler sonography (CCDS) and artifact-optimized imaging in high-resolution (HR) mode and with the option of glazing with microflow flow methods additionally adapted to low flow as short cine loops and with single frames. All new flow options were available under function UMA. A wheel spoke pattern was considered typical for focal nodular hyperplasia (FNH).

The evaluation of the liver parenchyma with regard to echogenicity was performed in comparison to the healthiest possible kidney parenchyma and was measurable in this respect under the function hepatorenal index (HRI+) as an index with ideal values up to 1. With color-coded elastography, the shear wave velocity was to be measured in the area of circular, individually adjustable regions of interest (ROI) in kPa or m/s. In this case, values < 1.4 m/s were target values for healthy parenchyma. In addition, a focused measurement was performed at a depth of 2 to 4 cm from the capsule using the STQ technique, at least 10 measurements are acquired, if possible outside vessels, not at bile ducts and in respiratory arrest. For this purpose, a quality indicator of maximum 5 green stars was available for orientation. Values of 1.4 m/s to 2.6 m/s were considered indicative of increasing fibrosis from F1 to F4. Higher values were considered to be evidence of cirrhosis.

The article "Current aspects of multimodal ultrasound liver diagnostics using contrast-enhanced ultrasonography (CEUS), fat evaluation, fibrosis assessment, and perfusion analysis – An update" was retracted in 2025. Reasons: compromised peer review; concerns about the citations; concerns about a third party's involvement.

With 2 additional tools, the degree of possible steatosis could be measured with documentation of possible artifact overlay and assessment in Liver texture index (LTI) mode for additional possible inflammatory changes. All liver parenchyma measurements were performed at a depth of 1 to a maximum of 5 cm, if possible, without recording vascular structures while avoiding motion and respiratory artifacts. Overall, a summary evaluation was possible under the USAT function (USAT, LTI, HRI+).

For the fat measurements, up to 10 individual measurements were targeted. Ideal values were measurements up to 0.5 dB/cm/MHz. Values > 0.8 dB/cm/MHz were indicated of measured values of a clear steatosis.

Contrast enhanced ultrasonography (CEUS) was used to clarify non-cyst focal liver lesions. As a bolus of 1 to 2.4 ml i.v. of sulphur-hexafluoride microbubbles (SonoVuetrademark, Bracco, Italy) with bolus administration of 10 ml NaCL was injected via cubital CEUS, the main lesion to be assessed was examined digitally as cine loops in DICOM format with respect to microvascularization. Following a low mechanical index (MI) technique (MI < 0.15), low MI penetration depth was frequency adapted via general (GEN), resolution (RES) or penetration (PEN) function. Perfusion evaluation with false color due time intensity curve (TIC) analysis was then performed from the up to 60 s capturing approach with onset of possible wash out in the early portal venous phase.

Parametrically, 10 s from the arterial insufflation were coded in false colors. Red and orange imply strongly hyper-vascularized portions, yellow moderate perfusion, green and blue low. A regular pattern typically appears in benign lesions, such as nodular from the margin in hemangiomas, homogeneous in fat distribution disorders, radicular from the center in FNH, from margin to center in adenomas. The main criteria for characterization of malignant lesions were irregular arterial microvascularization in CEUS, almost too chaotic pattern in HCC, and wash out increasing to late phase from 3 to 5 min. These wash out kinetics were recorded with short cine loops of 10 s over the entire liver every 60 s if possible.

The article "Current aspects of multimodal ultrasound liver diagnostics using contrast-enhanced ultrasonography (CEUS), fat evaluation, fibrosis assessment, and perfusion analysis – An update" was retracted in 2025. Reasons: compromised peer review; concerns about the citations; concerns about a third party's involvement.

Measurement parameters of the TIC analysis were time to peak (TTP), peak enhancement, mean transit time (mTT) and area under the curve (AUC). These can be stored in a protocol. Benign changes typically demonstrate a rather continuous increase of the contrast enhancement of the lesion until it is aligned with the surrounding area. Malignant lesion exhibits micro shunts with irregular hypervascularization, rapid curve rises and then wash out with curve flattening. Post ablation defects or scars after tumor resection should be avascular.

### 2.1 Low-velocity microvascular blood flow-Ultra Micro Angiography (UMA)

The ultrasound microvascular real-time imaging was established using a novel technology of the Mindray Resona R9 ultrasound imaging platform. Benefitting from the CPU/GPU processing performance of the Resona R9 platform, UMA acquires high-quality raw ultrasonic signals through the ultrasonic plane wave/divergent wave (hereinafter referred to as plane wave) at high efficiency and utilizes an advanced tissue-rejection algorithm to intelligently remove tissue clutter from raw signals. These two core techniques allow UMA to break through the technical bottleneck of traditional Color Doppler Flow Imaging, that greatly improving the sensitivity and spatial resolution of blood flow detection, and visualizes microvascular architecture undetectable by traditional CDFI.

### 2.2 UltraSound ATtenuation imaging technology (USAT)

USAT provides a new and easy tool that obtains ultrasound attenuation imaging and measurement to diagnose fatty liver quantitatively. Based on the innovative “Full Space Restitution Technology”, USAT restitutes the real sound speed and attenuation from ultrasonic echoes improving accuracy and reproducibility of measurements. Accurate quality control indicators help users obtain higher quality ultrasound attenuation images and measurements. Flexible and convenient research tools allow a user to conduct clinical studies for various purposes, such as screening, diagnosis, and follow-up of fatty liver disease.

USAT provides good consistency with steatosis grading based on B-mode imaging, demonstrating its great potential to determine the stages of fatty liver disease, as shown in the figure below, the mean values of USAT in different steatosis grades based on B-mode imaging were 0.49, 0.59, 0.70, and 0.90 dB/cm/MHz respectively. It can be seen that USAT measurements increase with the progression of fatty liver disease. Steatosis was categorized based on Brunt grading as follows: S0 < 5%, S1 = 5% –33%, S2 = 34% –66% and S3≥67%. The recommend cutoff value of USAT are 0.53, 0.66, 0.82 dB/cm/MHz respectively.

The article "Current aspects of multimodal ultrasound liver diagnostics using contrast-enhanced ultrasonography (CEUS), fat evaluation, fibrosis assessment, and perfusion analysis – An update" was retracted in 2025. Reasons: compromised peer review; concerns about the citations; concerns about a third party's involvement.

### 2.3 ZONE sonography technology plus (ZST+) technology (high frame rate HiFR CEUS)

The ZST + technology adopts the weak focused transmission, generating wider physical beams. The area scanned in each transmission is significantly larger than that in traditional focused transmission. The plane wave technology applies the non-focused whole-zone transmission mode. The entire imaging area is scanned in one transmission. Therefore, one frame of image can be generated with one transmission. In addition, due to the weak focused transmission and non-focused transmission modes, both two zone transmission technologies require post processing at the receive end, to achieve a higher frame rate without compromising the image quality of the contrast imaging. For focused imaging, the lateral resolution and signal-to-noise ratio (SNR) of the sound field at the focus are the best, but the performance is gradually degraded away from the focus. The lateral resolution of the entire field can be improved by increasing the number of transmission foci or adopting continuous focused transmission at the cost of an inevitably decreased frame rate. This is infeasible for the focused imaging with a low upper limit of the frame rate. Although the overall lateral resolution is poorer than that at the focus of the focused transmission, the sound field is more uniform. With the reconstruction of the receiving sound field, the continuous transmission focused synthetic sound field could be achieved. In addition, with the coherent transmission synthesis technology, the number of transmissions is significantly reduced. Furthermore, in order to tackle the problem of line artifact and SNR loss caused by decreased transmissions, each receiving line is generated through optimized compounding of echoes from adjacent multiple transmissions. To sum up, the ZST + technology is the key to HiFR-CEUS by increasing the frame rate of CEUS without compromising image quality.

HiFR-CEUS was performed in bolus technique as intravenous administration of 1–2.4 ml Sulphur hexafluoride microbubbles contrast agent SonoVuetrademark with 10 ml NaCL (saline solution) via cubital vein [23]. Possible history of contrast intolerance was considered a contraindication. Impaired renal function or renal insufficiency or changes in thyroid function were not considered contraindications according to the EFSUMB guidelines [10]. The examinations were performed dynamically with the new HiFR technique depth-adapted with the modalities GEN, RES or PEN and digitally documented. The CEUS examinations of the entire liver performed in sweep technique included continuous acquisition of the arterial phase 10 to 15 s after bolus administration to the portal venous phase over 1 minute, in case of vascular changes with optimal acquisition of the hepatic hilus to be able to detect possible arteriovenous or portal venous macro- or micro shunts. Then, lesion- and findings-related documentation of a possible wash-out was performed with short cine loops over 5 to 10 s up to a late phase of 5 to 6 minutes, supplemented by single images that could be stored during the cine sequences specifically related to findings. The images were automatically sent to PACS for independent analysis.

The article "Current aspects of multimodal ultrasound liver diagnostics using contrast-enhanced ultrasonography (CEUS), fat evaluation, fibrosis assessment, and perfusion analysis – An update" was retracted in 2025. Reasons: compromised peer review; concerns about the citations; concerns about a third party's involvement.

## 3 Results

In 47/50 cases, a final assessment was possible with multimodal ultrasound diagnostics. In 3 cases with suspected HCC, ultrasound-guided biopsy was performed additionally for final diagnosis.

In all 25 cases of malignant liver lesions and in postoperative defects or after tumor ablation, complementary cross-sectional imaging with contrast-enhanced multiphase computed tomography (CT) and or magnetic resonance imaging (MRI) with liver-specific contrast agent (Primovisttrademark, Bayer, Germany) was performed according to the guidelines of the tumor board to validate the findings.

The diagnosis of different degrees of fatty liver by USAT (38/50 cases) and a degree of fibrosis with STQ F1 to F4 according to Colombo (32/50 cases) was validated by follow-up in all cases. Ultrasound-guided biopsy was performed in 9 cases. In B-scan morphological criteria of cirrhosis, only fibrosis grade F3 was found in 3 cases with corresponding changes also in magnetic resonance imaging (MRI) (Fig. 1).

**Fig. 1:** New ultrasound modalities of non-invasive evaluation of the liver stiffness in a case of F1 fibrosis up to 1.5 m/s (a), color-coded shear wave technique with high image quality (5 green stars) with blue and less yellow colors parts as a sign of less liver stiffness (b). Using the new liver tissue technologies the parenchymal comparison from kidney cortex and liver tissue is possible with values > 1,2 (HRI+) and values up to 0.7 dB/cm/MHz for the liver fatty measurements (USAT) (c). LTI measurements with values up to 3.8 after chronic inflammatory reaction (d). High image quality of 100% and 5 stars in all case (e).

Improved flow detection using UMA in combination with HR flow and glazing flow allowed artifact-free flow detection in 5/50 cases after older near-echo portal vein thrombosis with proportionate signs of cavernous transformation (Fig. 2).

The article "Current aspects of multimodal ultrasound liver diagnostics using contrast-enhanced ultrasonography (CEUS), fat evaluation, fibrosis assessment, and perfusion analysis – An update" was retracted in 2025. Reasons: compromised peer review; concerns about the citations; concerns about a third party's involvement.

**Fig. 2:** Evaluation the liver vascularization after liver transplantation (LTX). Using the UMA technology simultaneous color coded flow evaluation of the hepatic artery, portal vein and the liver veins is possible (a). The new flow modalities enables with high quality the simultaneous detection of the low flow of the liver veins up to high flow of the hepatic artery (b).

Using HiFR CEUS (Fig. 3) and CEUS parametric and TIC analysis, independent evaluation confirmed the diagnosis of benign liver tumors in 25 cases, as malignant lesion in 9 cases with specific diagnosis in 6 cases (Fig. 4), as post-ablation defects after percutaneous treatment of previously malignant lesion in 11 cases and postoperative defects for follow-up in 5 cases (Fig. 5).

**Fig. 3:** A hypoechogenic solid lesion in the center of the liver (a). Using CEUS perfusion imaging by parametric false colors and TIC-Analysis detection of irregular tumor neo-vascularisation is possible (b). Considering the inhomogeneous liver tissue change this is typical for a hepatocellular carcinoma (LI-RADS V).

**Fig. 4:** Possibilities of parametric evaluation of dynamic CEUS by false colors of dynamic arterial microvascularization of the liver. By red color detection of early enhancement of vascular structures (a) and hyperenhancement of a tumor lesion by red, orange and yellow color maps, not detectable by the fundamental B-mode (b).

**Fig. 5:** CEUS perfusion imaging after complete treatments of malignant liver lesions by microwave ablation therapy (MWA). Parametric imaging using color maps could visualize the different perfusion parameters (AUC, PKI, WiAUC, AT) (a). TIC analysis shows not relevant enhancement in the center of the MWA defect (red) and continuous enhancement of the margin (yellow) and the liver tissue (blue) (b).

Among the 25 benign cases, 9 patients were found to have mildly echogenic foci compatible with FNH, 7 cases were echogenic with hemangiomas, 5 cases were of mixed echogenicities with regenerating nodules, 4 cases were echogenic lobulated segmental fat distribution disorders, and 1 patient was found to have a proportionally echogenic adenoma.

Of the 9 cases of malignant lesions, 3 cases were HCC, 1 was CCC, and 5 were colorectal liver metastases. In addition, 11 cases underwent control after microwave ablation (MWA) of originally malignant liver lesions (8 cases of HCC, 1 case of CCC, 2 cases of metastasis) and 5 cases underwent postoperative control (2 cases of HCC, 3 cases of colorectal metastasis).

Typically, benign lesions showed a regular vascular pattern with increasing contrast enhancement toward the late phase, whereas malignant lesions showed irregular arterial hypervascularization with wash out beginning in the portal venous phase.

The article "Current aspects of multimodal ultrasound liver diagnostics using contrast-enhanced ultrasonography (CEUS), fat evaluation, fibrosis assessment, and perfusion analysis – An update" was retracted in 2025. Reasons: compromised peer review; concerns about the citations; concerns about a third party's involvement.

In the parametric false colors, hypervascularization was coded orange to red, inferior perfusion was coded blue to green, and intermediate perfusion was coded yellow (Fig. 6).

The main limitations of TIC analysis were respiratory artifacts and deep lesions with a penetration depth of at least 12 cm [3] (Fig. 7). Due to more difficult sonic conditions in obesity and meteorism, or in pronounced ascites and cirrhosis, measurements for fibrosis and CEUS examinations at depth are sometimes of limited value.

**Fig. 6:** High resolution CEUS, parametric color coded imaging and CEUS perfusion imaging (a) with color maps of different perfusion parameters (DS, SR, FIT, mTT) and time intensity curve in a case of Osler's disease (b). Dynamic evaluation of the capillary microvascularization shows capillary shunts with early enhancement after 12 s, short mean transit time (MTT) and strongly global enhancement evaluated by the time-intensity-curve (TIC) (c).

**Fig. 7:** Color coded parametric and time intensity curve analysis (TIC) of dynamic microvascularization of a benign liver lesion using HiFR CEUS. Typical for a focal nodular hyperplasia (FNH) is the continuous enhancement for the center to the margin with than similar contrast like the live tissue. Color maps could visualize different perfusion parameters (AUC, PKI, WiAUC, AT).

## 4 Discussion

Multimodal ultrasound imaging of the liver with high-resolution B-mode technique, artifact-reduced vascular ultrasound, fibrosis measurement, fat evaluation, CEUS, and perfusion imaging poses new challenges even to experienced investigators. Already in own preliminary studies it could be shown that flow optimization by means of HR-flow and glazing flow can be very helpful in the acquisition of flow hemodynamics especially in difficult sonic conditions [24, 25], in cirrhosis with reduced portal vein flow and arterial collaterals [24, 25] in venous thrombosis and after transjugular intrahepatic portosystemic shunts (TIPS) installation [24, 25]. Flow techniques adapted even further to microflow are increasingly enabling better imaging of tumorous vascular patterns. For example, a spoke wheel pattern typical for FNH.

Nevertheless, dynamic acquisition of microvascularization using SonoVuetrademark as a strictly vascular ultrasound contrast agent leaves the assessment of dynamic tumor microvascularization to high resolution techniques of CEUS such as HiFR [3, 17]. The extent to which this can lead to an improved diagnosis of hepatocellular carcinoma (HCC) will be investigated in a multicenter study. Cholangiocellular carcinoma (CCC) can present similarly, but usually shows different wash out kinetics, for which CEUS perfusion evaluation is helpful [1].

The article "Current aspects of multimodal ultrasound liver diagnostics using contrast-enhanced ultrasonography (CEUS), fat evaluation, fibrosis assessment, and perfusion analysis – An update" was retracted in 2025. Reasons: compromised peer review; concerns about the citations; concerns about a third party's involvement.

At least preliminary studies indicate an improved characterization of differently pronounced peri-tumoral microvascularization with high-resolution contrast imaging in CEUS supplemented by parametric false-color imaging [2]. According to the Liver Imaging Reporting and Data System (LI-RADS) classification, the detection of small tumor foci in only arterial hypercontrast up to 10 mm, a reliable differentiation of adenomas or regressively altered tumors, and the detection of all tumor foci in poor acoustic conditions may require complementary imaging with CT and or MERT with liver-specific contrast agent as an alternative to histologic confirmation [26].

Increasingly, developments are being made that allow the tissue to be characterized in terms of capillary blood flow and tissue morphology with a high degree of detail. The increasingly rapid acquisition of measured values, especially with STQ analysis, makes it possible to record the degree of fibrosis up to cirrhosis more quickly, thus also facilitating progress monitoring. However, even with the additional color-coded display, the different measurement ranges of different device technologies are still a point of criticism of the sole shear wave evaluation.

Likewise, measurement ranges still need to be defined for recording the degree of liver fatty degeneration [6, 8, 27–29], although graduation at values up to 0.6 dB/cm/MHz, medium and clear at then values greater than 0.7 dB/cm/MHz proved reproducible. The comparison between liver parenchyma and renal parenchyma, now mapped in an index clearly depends on the sonic conditions into the retroperitoneum and on the morphology of the renal parenchyma. An apparently ideal value of 1 can also be obtained when both parenchyma of the liver and kidney are echo-rich altered, as in steatosis and drug toxic alteration of the kidney. In the case of hepatitis or cirrhosis, the additional LTI value to be measured can give an indication of the extent to which reactive inflammatory changes or interstitial edema are still present [30]. Malignant tumors can also lead to an increase in values [31–33]. CEUS parametric and with TIC analysis offers a very high diagnostic potential for a comprehensive analysis of tumor neoangiogenesis, especially with integrated software [3, 16–18, 34–36]. This opens up a multitude of application possibilities for therapy monitoring [35, 37–40]. Also, in own studies an improved postinterventional control by CEUS perfusion could be achieved with so far external perfusion software [16, 30, 32, 33, 35, 39–42]. Chemotherapy and chemoembolization (TACE) can also be monitored by CEUS perfusion [38, 39, 42]. This can be extended beyond the liver to other organs such as thyroid, lymph nodes, intestine, kidney and prostate. Further studies are needed for this.

The article "Current aspects of multimodal ultrasound liver diagnostics using contrast-enhanced ultrasonography (CEUS), fat evaluation, fibrosis assessment, and perfusion analysis – An update" was retracted in 2025. Reasons: compromised peer review; concerns about the citations; concerns about a third party's involvement.

## 5 Conclusion

State-of-the-art high-resolution technologies help to increase ultrasound diagnostic capabilities of liver cancers, especially in difficult cases. CEUS parametric and with TIC analysis opens up a new era for application for therapy monitoring.
